# The Effects of Periarticular Injection Cocktail in Postoperative Analgesia after Bilateral Unicompartmental Knee Arthroplasty

This article has been retracted.

**DOI:** 10.1155/2022/9289904

**Published:** 2022-07-28

**Authors:** Ruizhu Wang, Jin Zhao, Xiaojing Guo, Binping Ji

**Affiliations:** ^1^Department of Orthopaedics, Shanxi Huajin Orthopaedic Hospital, Taiyuan, Shanxi 030400, China; ^2^Department of Hematology, Shanxi Province Cancer Hospital/ Shanxi Hospital Affiliated to Cancer Hospital, Chinese Academy of Medical Sciences/Cancer Hospital Affiliated to Shanxi Medical University, Taiyuan, Shanxi 030013, China

## Abstract

**Objective:**

This study was conducted to compare postoperative pain and functional recovery in bilateral unicompartmental knee arthroplasty (UKA) and unilateral UKA after cocktail therapy.

**Methods:**

A total of 240 patients who received unilateral UKA and bilateral UKA in our orthopedic department from February 2019 to April 2020 were collected. The general clinical data was recorded and compared between the two groups of subjects, and the time of postoperative landing was recorded separately for both groups. A visual analogue scale (VAS) was used to record the patients' pain at 1, 7, and 14 days postoperatively, as well as the range of motion of the affected limb at 1, 7, 14 days, and 3 months postoperatively and the hospital for special surgery (HSS) knee score of the knee at 1 month postoperatively.

**Results:**

After cocktail injection analgesia, unilateral patients with knee surgery got off the ground and walked significantly earlier than patients with bilateral surgery, while there was no significant difference between the two groups in terms of pain at 1, 7, and 14 days after surgery, range of motion of the affected limb at 1, 7, 14 days, and 3 months after surgery, and knee HSS score at 1 month after surgery.

**Conclusion:**

Periarticular cocktail injection significantly reduces postoperative pain in patients, and bilateral UKA surgery can be used as satisfactory as unilateral UKA in clinical practice.

## 1. Introduction

Unicompartmental knee arthroplasty (UKA) and total knee arthroplasty (TKA) have been widely used in clinical treatment since the 1960s and 1970s [1]. It was gradually carried out in China around 2000 [2]. Because UKA is characterized by less surgical trauma, short operation time and less perioperative blood loss [3, 4], better restoration of native knee kinematics, and earlier restoration of gait [5], simultaneous replacement of double knee joints becomes safe and reliable. Atar et al. [6] compared and analyzed the treatment effects of 30 patients with UKA and 30 patients with TKA. The results showed that compared with UKA group, the incidence of postoperative rehabilitation and complications in TKA group was significantly higher. After 6 months of treatment, the total working extension value and flexion of knee joint in UKA group were significantly higher than those in TKA group. Sershon et al. [7] found that patients treated with UKA had shorter hospital stay and greater range of early knee movement, and short-term complications may be more common in TKA. The implementation of the double-side single condylar knee arthroplasty can effectively reduce the patient's bleeding and hospital stay and less postoperative morbidity [8, 9]. UKA allows patients to return to function more quickly than TKA, but postoperative pain management remains a challenge because there is no significant difference in pain [10, 11].

Cocktail injection analgesia mainly refers to the mixed local anesthetics (mainly ropivacaine, bupivacaine, glucocorticoid, morphine, etc.) and injecting them around the joints by local infiltration anesthesia (LIA) technology to play the role of postoperative analgesia [12]. Cocktail injection anesthesia has been widely used in clinical practice, and studies have shown that this method is ideal for analgesia in TKA [13], rhinoplasty [14], and spinal fusion [15]. A meta-analysis by Li et al. [16], on the efficacy of multimodal cocktail periarticular injections with additional corticosteroids in TKA, showed that multimodal cocktail periarticular injections with glucocorticoids reduced the intensity of early resting pain and increased early knee mobility after knee arthroplasty. The above study confirms that cocktail therapy is indeed effective in controlling postoperative pain and achieving good postoperative results. At present, there are few studies on the clinical efficacy of cocktail injection analgesia in postoperative analgesia after bilateral UKA. Therefore, in this study, we mainly investigated the analgesic effect of cocktail injection in bilateral UKA to provide more evidence-based medical evidence for the use of cocktail analgesia in clinical practice.

## 2. Materials and Methods

### 2.1. Patients

This study was a prospective controlled trial. A total of 240 patients who underwent primary UKA at Shanxi Hua Jin Orthopaedic Hospital from February 2019 to April 2020 were enrolled. This study was approved by the Ethics Committee of Shanxi Huajin Orthopaedic Hospital (2019003).

After screening, 120 patients who received bilateral UKA were in group 1. 120 patients who received unilateral UKA were in group 2. All surgeries were performed by the same group of senior doctors.

Inclusion criteria are as follows: (1) the affected knee joint lesions were limited to the medial compartment; (2) standing radiographs showed bone-to-bone wear in the diseased knee space; (3) the ligament function of the affected knee joint was good; (4) the varus deformity of the affected knee joint can be corrected; and (5) the patient had a clear desire for surgery and could cooperate with the whole study. Exclusion criteria are as follows: (1) patients with prior intolerance to the drugs involved in this study; (2) the patient has a history of dependence on analgesic drugs, alcohol, opioids, and other substances; and (3) patients who could not tolerate UKA after analysis of clinical examination results.

### 2.2. Operation Method

All patients were treated with general anesthesia and femoral nerve block anesthesia. During the operation, a tourniquet was routinely applied to the affected limb and the pressure was set at 350 mmHg. In the bilateral UKA group, the patients were operated on the side knee, which the patients thought was more painful. After the prosthesis was installed, the first assistant and the third assistant were sutured, and the operator and the second assistant were operated on the other side. The Oxford biotype monondylar prosthesis (Bomex) was selected as knee prosthesis in this study. The drainage tube was routinely indwelled and removed 24 hours after surgery. After surgery, postoperative rehabilitation team doctor to arrange the same rehabilitation guidance, and guide the patient after patient operation the quadriceps muscle and began to practice isometric contraction, pull out area after indwelling drainage tube began to conduct activities of knee joint flexion and extension and assisted the straight leg-raising practice, and to guide the patient down stand up under protection, and use a walker began walking practice.

### 2.3. The Analgesia Method of Cocktail Drug

The cocktail drug formulation was selected as follows: ropivacaine injection 300 mg (Guangdong Jiabo Pharmaceutical Co., LTD.), ketorolac 30 mg (Shandong Qilu Pharmaceutical Co., LTD.), and epineadrenaline 1 mg (Shandong Qilu Pharmaceutical Co., LTD.), diluted with 0.9% sodium chloride solution for 50 ml. Cocktail medicine injection is the way both for multipoint infiltration in articular cavity injection, injection point selection for the back of the joint capsule, the quadriceps tendon, patellar ligament around organization, shin fat pad, incision fat, and subcutaneous tissue, before each injection time for knee joint prosthesis placed articular cavity flushing after injection amount to 50 ml of drug cocktail each knee.

### 2.4. Observation Indicators

The time for patients to go to the ground after surgery was recorded. Patients' pain assessment of was recorded on 1, 7, and 14 days after surgery. The visual analogue scale (VAS) was selected as the pain scoring standard, and the range of motion of patients' affected limbs on 1, 7, 14 days, and 3 months after surgery was recorded. The hospital for special surgery (HSS) knee score was evaluated one month after surgery.

### 2.5. Statistical Analysis

The SPSS19.0 statistical software was used to process the experimental data. The measurement data involved were expressed as mean ± standard deviation (SD), and *t*-test was adopted. The counting data was expressed as number, and chi-square test was used. *P* < 0.05 indicated a statistically significant difference.

## 3. Results

### 3.1. General Clinical Information

A total of 240 patients from February 2019 to August 2019 met the inclusion criteria, with 120 patients in each of the two groups. Patients in group 1 had unilateral UKA (male 26, female 94), and group 2 had bilateral UKA (male 25, female 95). The gender, age, weight, and height of the patients in the two groups were compared separately, and the differences were not statistically significant, which proved that the two groups were comparable (Table 1).

### 3.2. Patients' Underground Time

As can be seen in Table 2, the between-landing time after surgery was 27 ± 8.44 h for group 1 and 22 ± 6.31 h for group 2, and group 1 was significantly lower than group 2 (*P* < 0.05). The data indicated that patients in the unilateral UKA group had earlier postoperative ground movement time.

### 3.3. Assessment of Patients' Pain after Surgery

No significant statistical difference was found between the two groups on the 1st, 7th, and 14th days after surgery, as shown in Table 3. It indicated that there was no difference in pain assessment between the two groups on the 1st, 7th, and 14th days after surgery. These results showed that cocktail injection around the joint cavity during surgery could effectively improve the postoperative pain of patients, and the same pain control effect can be achieved in patients undergoing unilateral and bilateral UKA.

### 3.4. Knee Function Assessment 1 Month after Surgery

There was no significant difference in the range of motion of the affected limb between the two groups on the 1st, 7th, 14th days, and the 3rd month after surgery, indicating that the injection of cocktail drugs around the joint during surgery was effective in pain control, and the range of motion of the knee joint in the two groups also achieved the same effect. One month after surgery, the HSS scores of patients in group 1 and group 2 were 95.57 ± 2.44 and 94.92 ± 1.92, with no significant statistical difference (*P* = 0.863). There was no difference in knee function between the two groups one month after surgery (Table 4). These results suggest that unilateral and bilateral single-condyle replacement can achieve the same therapeutic effect one month after operation with injection of periarticular cocktail of analgesic drugs and rehabilitation therapy.

## 4. Discussion

As the ultimate treatment for knee osteoarthritis, knee replacement has been widely carried out globally with the number of hundreds of thousands of operations per year [2]. With the continuous progress of surgical technology and perioperative management concept, the enhanced recovery after surgery (ERAS) concept has gradually penetrated into the clinical application of relevant surgical departments and departments. Compared with TKA, UKA has shorter operation time, less surgical trauma, shorter operation, and anesthesia time, all of which conform to the promotion of ERAS concept [2, 4]. Leiss et al. [11] compared the parameters after performing a 1 : 1 matched pair analysis, multicenter-wide in 14 orthopedic departments. Pain scores were significantly lower for the UKA group than those for the TKA group. In the recovery unit, there was less need for pain medication in patients with UKA. The opiate consumption was similarly lower for the UKA group, but not statistically significant. In the ward, the UKA group needed less opioids. This shows that UKA has more advantages.

However, pain after knee replacement has always been an important factor of restricting knee replacement effect [17], lived around joints in knee surgery is a cocktail drugs can effectively alleviate postoperative pain, and is compared with femoral nerve block and vertebral canal or intravenous patient controlled analgesia, has little influence on quadriceps, benefit patients early postoperative activities, avoid wrestling and reduce opioid nausea, lethargy and other adverse reactions [18, 19]. When choosing a drug cocktail, different joint surgeons take different drug cocktail formulations for different reasons. In this study, ropivacaine was used as a local anesthetic, mainly on the basis of ropivacaine's advantages of sensory and motor nerve separation and less influence on postoperative movement, and compared with other local anesthetics, ropivacaine also has advantages of low cardiac and central toxicity and long acting time [20]. A series of studies have shown that its analgesic effect in ophthalmic surgery, dental surgery, and obstetrical and gynecological surgery is superior to that of other anesthetic drugs [21–24]. Ketorolac is a nonsteroidal anti-inflammatory and analgesic drug that can exert analgesic effects by inhibiting the production of inflammatory pain-causing transmitters. With the assistance of adrenaline, ropivacaine and ketorolac can exert effect in the surrounding tissues of the operation area for a long time and reduce the pain of patients [25].

Our findings showed a significant difference in time to first postoperative flooring between the two groups, with those who underwent unilateral UKA having an earlier flooring time than those who underwent unilateral UKA, which is consistent with previous findings by Suleiman et al. [26] in a related study comparing bilateral and unilateral total knee arthroplasty. The safety of simultaneous bilateral total knee arthroplasty has been controversial; in a study comparing the complications and mortality associated with surgery in the hands of 629 female TKA patients (308 SBTKA and 321 UTKA) in Korea, the results showed that the SBTKA group had a significantly higher incidence of postoperative confusion and hypoxia during hospitalization and a longer hospital stay, but there was no difference in the incidence of serious postoperative complications (such as myocardial infarction and deep vein thrombosis) between the groups during hospitalization. There was no difference in the incidence of serious postoperative complications (e.g., myocardial infarction and deep vein thrombosis) between the groups during hospitalization, and at six months, there were no procedure-related deaths in either group, suggesting a fair safety profile for simultaneous bilateral knee surgery [27]. A retrospective study by Ahn et al. [28] showed fewer perioperative complications, less bleeding, fewer transfusions, and better functional outcomes 6 months after bilateral simultaneous UKA compared to unilateral TKA. In this study, we found no significant difference in pain levels between patients undergoing bilateral simultaneous UKA surgery and unilateral surgery, indicating that intraoperative injection of a cocktail of drugs around the joint can effectively relieve patients' pain conditions. It does not increase the risks associated with surgery. It was also found that there was no significant difference in the knee HSS scores between the two groups at 1 month postoperatively, indicating that the use of cocktail analgesia during simultaneous bilateral UKA surgery did not increase the time to recovery of limb function after surgery, which again validates the efficacy and safety of this method in bilateral UKA surgery.

Cocktail therapy applied to joint surgery has been widely used in the last two decades, and different surgeons have gained a lot of experience in clinical work [12, 29, 30]. However, it is still in the position of selecting drugs with the main purpose of controlling pain and reducing bleeding. Some studies have suggested that the addition of hormones such as dexamethasone to the formulation can reduce postoperative adverse effects [19, 31], but the effectiveness remains to be further clinically observed. In the long run, cocktail therapy still has a more promising future.

The strength of this study is that it has a sufficient sample size to have some persuasive statistical inference. The limitation is that the trial design did not include a blank control, and the cocktail ratios were not set differently, so it is impossible to determine whether the ratios in this study are the best ratios for analgesia in patients with bilateral UKA.

## 5. Conclusion

In summary, periarticular injection cocktail analgesia has no significant adverse experiential stimuli for patients undergoing bilateral UKA surgery, and both can be actively involved in subsequent rehabilitation practices and related treatments with satisfactory therapeutic outcomes.

## Figures and Tables

**Table 1:** Demographic characteristics.

Features	Group 1 (*n* = 120)	Group 2 (*n* = 120)	*P*
Gender (male/female, *N*)	26/94	25/95	0.903
Age (years)	63.46 ± 9.22	62.75 ± 8.39	0.147
Weight (kg)	59.56 ± 7.42	61.04 ± 8.64	0.281
Height (cm)	156.34 ± 11.20	155.81 ± 9.31	0.491

Data was expressed as *n* or mean ± SD. Group 1: patients received bilateral unicompartmental knee arthroplasty (UKA). Group 2: patients received unilateral UKA.

**Table 2:** Comparison of the underground time between the two groups.

Features	Group 1 (*n* = 120)	Group 2 (*n* = 120)	*P*
Time, hours	27 ± 8.44	22 ± 6.31	0.031

**Table 3:** Comparison of pain (visual analogue scale) between the two groups.

Time	Group 1 (*n* = 120)	Group 2 (*n* = 120)	*P*
Postoperative 1 day	5.36 ± 1.93	5.24 ± 2.04	0.062
Postoperative 3 days	3.13 ± 1.41	3.16 ± 1.58	0.083
Postoperative 7 days	2.34 ± 1.25	2.30 ± 1.31	0.077

**Table 4:** Knee function assessment (HSS scores) between the two groups.

Time	Group 1 (*n* = 120)	Group 1 (*n* = 120)	*P*
Postoperative 1 day	35.36 ± 11.7	38.41 ± 15.0	0.291
Postoperative 3 days	53.26 ± 12.43	55.79 ± 11.82	0.449
Postoperative 7 days	92.34 ± 7.64	91.30 ± 8.31	0.672
Postoperative 1 months	95.57 ± 2.44	94.92 ± 1.92	0.7863
Postoperative 3 months	125 ± 11.82	131 ± 14.77	0.773

## Data Availability

The data used to support the findings of this study are available from the corresponding author upon request.
